This article has been retracted.

# Regulation of DNA Repair Mechanism in Human Glioma Xenograft Cells both *In Vitro* and *In Vivo* in Nude Mice

**DOI:** 10.1371/journal.pone.0026191

**Published:** 2011-10-14

**Authors:** Shivani Ponnala, Krishna Kumar Veeravalli, Chandramu Chetty, Dzung H. Dinh, Jasti S. Rao

**Affiliations:** 1 Department of Cancer Biology and Pharmacology, University of Illinois College of Medicine at Peoria, Peoria, Illinois, United States of America; 2 Department Neurosurgery, University of Illinois College of Medicine at Peoria, Peoria, Illinois, United States of America; Johns Hopkins Hospital, United States of America

## Abstract

**Background:**

Glioblastoma Multiforme (GBM) is the most lethal form of brain tumor. Efficient DNA repair and anti-apoptotic mechanisms are making glioma treatment difficult. Proteases such as MMP9, cathepsin B and urokinase plasminogen activator receptor (uPAR) are over expressed in gliomas and contribute to enhanced cancer cell proliferation. Non-homologous end joining (NHEJ) repair mechanism plays a major role in double strand break (DSB) repair in mammalian cells.

**Methodology/Principal Findings:**

Here we show that silencing MMP9 in combination with uPAR/cathepsin B effects NHEJ repair machinery. Expression of DNA PKcs and Ku70/80 at both mRNA and protein levels in MMP9-uPAR (pMU) and MMP9-cathepsin B (pMC) shRNA-treated glioma xenograft cells were reduced. FACS analysis showed an increase in apoptotic peak and proliferation assays revealed a significant reduction in the cell population in pMU- and pMC-treated cells compared to untreated cells. We hypothesized that reduced NHEJ repair led to DSBs accumulation in pMU- and pMC-treated cells, thereby initiating cell death. This hypothesis was confirmed by reduced Ku70/Ku80 protein binding to DSB, increased comet tail length and elevated γH2AX expression in treated cells compared to control. Immunoprecipitation analysis showed that EGFR-mediated lowered DNA PK activity in treated cells compared to controls. Treatment with pMU and pMC shRNA reduced the expression of DNA PKcs and ATM, and elevated γH2AX levels in xenograft implanted nude mice. Glioma cells exposed to hypoxia and irradiation showed DSB accumulation and apoptosis after pMU and pMC treatments compared to respective controls.

**Conclusion/Significance:**

Our results suggest that pMU and pMC shRNA reduce glioma proliferation by DSB accumulation and increase apoptosis under normoxia, hypoxia and in combination with irradiation. Considering the radio- and chemo-resistant cancers favored by hypoxia, our study provides important therapeutic potential of MMP9, uPAR and cathepsin B shRNA in the treatment of glioma from clinical stand point.

## Introduction

Glioblastoma Multiforme (GBM) is a highly malignant tumor of the central nervous system with a median survival rate of less than 12 months and with a high rate of recurrence. The genetic makeup of GBM is complex involving a number of chromosome aberrations and genetic alterations in several genes [1], [2]. Chromosomal double strand breaks (DSBs) caused by genomic instability are considered to be toxic DNA lesions compared to others [3]. Stabilization of irradiation (IR)-induced DNA damage usually fails not only due to an hypoxic environment but also by the enhanced DNA repair ability of glioma cells [4]. Efficiency of glioma cells to elevate DNA damage repair, anti-apoptotic mechanisms and other growth survival signaling pathways enhance GBM proliferation, and in addition to hypoxia make treatment of GBM difficult [5], [6].

DSBs can be repaired either by non-homologous end joining (NHEJ) or homologous recombination (HR). In mammalian cells, NHEJ is the predominant DSB repair mechanism compared to HR [7]. Both DNA protein kinase catalytic subunit (DNA PKcs) and ataxia talengiectasia mutated (ATM) belong to the phosphatidylinositol kinase family. The serine-threonine kinase activity of these proteins is involved in cellular functions such as DNA damage surveillance, transcription and cell cycle progression [8]. DNA PK comprising the DNA PKcs, Ku70 and Ku80, form complexes at DSBs to initiate repair by NHEJ mechanism. Proficient repair of DSBs has been associated with over-expression of DNA PKcs [9]. ATM plays an important role in DNA damage response (DDR) by facilitating cell cycle arrest or triggering apoptosis based on the severity of the damage [10]. Growth signaling proteins such as Epidermal growth factor receptor (EGFR) are over-expressed in various cancers including GBM [11], [12]. EGFR is shown to physically interact with DNA PK and regulate its activity [13].

Earlier studies have shown the increased expression levels of matrix metalloprotease 9 (MMP9) and its correlation with the histological grade of glioma malignancy [14], [15]. Moreover, interaction of MMP9 with the Ku protein at the cell surface of leukemia cell lines was associated with cell invasion [16]. Urokinase-type plasminogen activator receptor (uPAR) expression is elevated in many human cancers including GBM and is indicative of poor prognosis [17]. Urokinase receptors have been shown to influence the expression of other proteases such as cathepsin B and MMP9, which are overexpressed in GBM [18], [19]. Furthermore, uPAR interaction with uPA has been shown to activate a downstream signal cascade involving plasminogen and MMP, which leads to ECM degradation, the release of growth factors, and ultimately tumor growth [20], [21]. Our earlier studies clearly demonstrated the efficacy of simultaneous downregulation of these bicistronic plasmid shRNA constructs in treating tumors by reducing adhesion, migration and invasion potential and inducing apoptosis in cancer cells [22]–[26]. However, none of our earlier studies have addressed the effect of these bicistronic constructs on DNA damage response (DDR) and the related molecular mechanisms involved. Hence, as the first step towards understanding the signal transduction in DDR in DSB repair, in the present study, we have used human glioma xenograft cells and treated them with MMP9+uPAR (pMU) and MMP9+cathepsin B (pMC) bicistronic plasmid shRNA constructs in both *in vitro* and *in vivo* models.

Here, we have demonstrated the role of MMP9 in combination with uPAR/cathepsin B in DDR in glioma xenograft cells. Our results clearly demonstrated that pMU and pMC treatments alter DNA repair efficiency, induces apoptosis and depletes survival signals in normoxic, hypoxic and hypoxic+IR exposed glioma cells.

## Results

### pMU and pMC treatments regulates non-homologous end joining (NHEJ) DNA repair proteins

NHEJ repair mechanism accounts for more than 75% of DSB repair in mammalian cells. To investigate the role of pMU and pMC treatments in DDR, we analyzed the expression of NHEJ related proteins DNA PKcs, Ku70 and Ku80. Our results showed reduced expressions of these proteins in pMU- and pMC-treated samples at both mRNA and protein levels in 4910 and 5310 cells (Figure 1A). We also observed that pDNA PKcs T2609 expression, a marker for NHEJ activation, was significantly reduced in pMU- and pMC-treated samples in these glioma cells (Figure 1A and 1B). We observed uPAR interaction with β1 integrin and co-immunoprecipitation of uPAR with MMP9 and cathepsin B (Figure 1C). We anticipate that these interactions among MMP9, uPAR, cathepsin B and β1 integrin demonstrate β1 integrin-mediated ECM signaling in reduced activity of NHEJ in pMU- and pMC-treated 4910 and 5310 glioma xenograft cells compared to untreated cells. Thus, pMU and pMC treatments in glioma xenograft cells play an important role in cellular signaling regulating the expression of NHEJ repair machinery.

**Figure 1:** Downregulation of non homologous end joining DNA repair machinery by pMU and pMC in glioma xenograft cells. A. RT PCR analysis showing expression of NHEJ related genes in pMU- and pMC-treated 4910 and 5310 glioma cells. GAPDH shows equal loading. Western blot analysis performed using cell lysates prepared from pMU and pMC silenced 4910 and 5310 glioma cells showing expression of DNA PKcs, pDNA PKcs, Ku70 and Ku80. GAPDH was analyzed as loading control. Each experiment was repeated 3 times. B. Further, quantification of the Western blots using ImageJ (NIH) software to determine the levels of these proteins after pMU and pMC treatments is shown. n = 3. Values shown are the mean (±SD). *p<0.05 vs. control. C. Immunoprecipitation (IP) analysis. IP of β1 integrin was immunoprobed with uPAR in both 4910 and 5310 glioma xenograft cells. IP of uPAR was immunoprobed with MMP9 and cathepsin B in glioma cells. Each experiment was repeated 3 times.

### pMU and pMC treatments inhibit proliferation of 4910 and 5310 glioma xenograft cells

In the present study, BrdU incorporation assay and survival fraction showed a significant decrease in the proliferation of 4910 and 5310 glioma cells treated with pMU and pMC compared to control and pSV-treated cells. Cell proliferation by BrdU assay showed a 45–50% reduced proliferation rate in pMU- and pMC-treated 4910 and 5310 glioma cells compared to control and pSV (Supplementary Figure S1A). Survival fraction from the clonogenic assay showed a 70–80% and 75–80% decrease in colony forming units after 2 weeks of pMU and pMC treatments respectively, compared to control and pSV-transfected cells (Supplementary Figure S1B). We have recently shown the efficiency of pMU and pMC constructs in downregulating respective target genes in treated 4910 and 5310 glioma xenograft cells [26].

### pMU and pMC treatments reduce EGFR-mediated DNA PK activity

EGFR expression plays an important role in proliferation and survival signals in cells [27]. EGFR interacts with DNA PK and regulates its activity [13]. As shown in Figures 2A and Supplementary Figure S1C, the expression of EGFR was decreased in pMU- and pMC-transfected glioma cells as compared to the controls. Perinuclear expression and nuclear internalization of EGFR is brought about by caveolin-1 (Cav-1). We observed the reduced expression of cav-1 (Figure 2A), integrin β1 and cSrc [26] in pMU- and pMC-transfected glioma cells compared with pSV and control. In addition, we investigated the interaction of EGFR with DNA PK by immunoprecipitation (IP) analysis. As shown in Figure 2B, IP of DNA PKcs and immunoprobed with EGFR showed reduced interaction with EGFR in pMU- and pMC-treated glioma cells compared to control and pSV-treated samples. Further, IP with EGFR and immunoblotting with Ku70 and Ku80 showed decreased association in pMU- and pMC-treated 5310 glioma xenograft cells compared to control (Figure 2B). In the present study, we evaluated the nuclear expression of these proteins. Figure 2C clearly showed that the nuclear expression of DNA PKcs, Ku70, Ku80 and EGFR was downregulated after pMU and pMC treatments. Moreover, the expression of SP1, a known transcription factor of DNA PKcs, Ku70 and Ku80, was reduced in pMU- and pMC-treated glioma cells compared to untreated cells (Figure 2A). Based on our results, it is very clear that there is a decreased activity of DNA PK, a key protein complex involved in initiation of NHEJ repair mechanism after pMU and pMC treatments in 4910 and 5310 glioma cells.

**Figure 2:** Regulation of DNA PK activity in pMU- and pMC-transfected glioma cells. A. Western blot analysis shows expression of EGFR, cav-1 and SP1 in pMU- and pMC-treated glioma cells along with control and pSV. B. Immunoprecipitation (IP) analysis. IP of DNA PKcs was immunoprobed with EGFR in both 4910 and 5310 glioma xenograft cells transfected with pMU and pMC along with control and pSV samples. IP of EGFR was immunoprobed with Ku70 and Ku80 in pMU and pMC treated glioma cells. IgG shows equal loading. C. Immunoblot analysis of DNA PKcs, Ku70, Ku80 and EGFR from nuclear lysates was carried out in pMU and pMC silenced 4910 and 5310 glioma xenograft cells. Lamin B was used for equal loading. Each experiment was repeated 3 times.

### pMU and pMC treatments inhibit Ku binding to DSBs and alters expression of DNA damage response (DDR) proteins

Ku70 and Ku80 binding efficiency to DSBs plays a major role in the initiation of NHEJ repair mechanism [7]. From our quantitative analysis of the efficiency of Ku70 and Ku80 binding to oligonucleotide, it is evident that the ability of Ku70 and Ku80 proteins to bind to the DSBs was significantly reduced in pMU- and pMC-treated samples in both 4910 and 5310 xenograft cells (Figure 3A). The binding of Ku70 to DNA was reduced by 50% in pMU-treated and 45% in pMC-treated 4910 glioma cells compared to controls. In addition, the binding of Ku80 was reduced by 58% in pMU and 50% in pMC-treated 4910 glioma cells compared with controls (Figure 3A). Similar results were observed in 5310 cells, wherein 60% and 46% of Ku70 and 39% and 37% of Ku80 binding to DNA were decreased in pMU- and pMC-treated samples, respectively, compared to controls (Figure 3A). This result indicates a reduction in the initiation of NHEJ repair in pMU- and pMC-treated glioma xenograft cells. These findings further strengthen our earlier findings wherein our pMU and pMC treatments lowered DNA PK activity in these glioma xenograft cells.

**Figure 3:** Inhibition of Ku activity and DDR related protein expression by pMU- and pMC-treated glioma xenograft cells. A. Ku70/80 DNA repair protein assay performed by using Active motif kit shows Ku70 and Ku80 protein binding to oligonucleotide in pMU- and pMC- treated 4910 and 5310 glioma xenograft cells along with control and pSV, respectively. Error bars indicate ±SD. * significant at p<0.05 Vs control. B. Immunoblot analysis showsexpression of key proteins involved in homologous recombination and DNA repair, such as ATM, pATM, RAD51, CHK2, pCHK2, ATR, pATR and pBRCA in both 4910 and 5310 glioma cells treated with pMU and pMC. Survival pathway protein such as ERK, pERK AKT and pAKT were analyzed using Western blot in pMU- and pMC-treated 4910 and 5310 glioma xenograft cells. Hypoxia assoaciated, HIF-1α expression was analyzed in both cell types after pMU and pMC treatments. GAPDH shows equal loading. C. Immunocytochemistry analysis was carried out to show co-localization of pATM and γH2AX foci in pMU- and pMC-treated 5310 glioma xenograft cells along with control and pSV. pATM expression can be visualized as red dots and γH2AX foci as green spots. Merged image shows co-localization as yellow to orange spots. Magnification 60×, Bar = 10 µm. Each experiment was repeated 3 times.

We also investigated the expression of proteins involved in homologous recombination (HR) and others such as ATR, pATR and pBRCA by Western blotting. As shown in Figure 3B, the expression of ATM, Rad51 and pCHK2 were downregulated in pMU- and pMC-treated glioma cells compared to control and pSV. In contrast, pATR expression was elevated in both 4910 and 5310 glioma cells with pMU and pMC treatments compared to controls (Figure 3B). ATM-mediated repair response to DSBs is initiated by its binding to DSBs. Co-localization studies of γH2AX foci and pATM showed reduced interaction in pMU- and pMC-treated 4910 and 5310 cells compared to control and pSV (Figure 3C). Pro-survival signals mediated by ERK and AKT were downregulated in pMU- and pMC-treated glioma cells as compared to untreated cells (Figure 3B). These results are consistent with earlier reported studies wherein inhibition of AKT and ERK impairs DNA repair in cancer [28], [29]. Hypoxia inducing factor – 1 alpha (HIF-1A), is markedly reduced in pMU- and pMC-transfected glioma cells compared to control samples (Figure 3B). Taken together, our results indicated a reduced HR repair in pMU- and pMC-treated 4910 and 5310 cells.

### pMU and pMC treatment results in DNA damage accumulation and apoptosis

Based on the aforementioned results, we hypothesized that reduced DDR in pMU- and pMC-treated glioma cells might result in accumulated damaged DNA. To test this hypothesis, we assessed accumulated DNA DSBs by comet assay. Comet tail length was increased in pMU- and pMC-treated glioma cells compared to control and pSV, indicating the accumulation of DSBs (Figure 4A). Figure 4B is a representative bar graph showing a significant increase in comet tail length in pMU- and pMC-treated 4910 and 5310 glioma cells.

**Figure 4:** Accumulation of double strand breaks in MU and MC knockdown 4910 and 5310 human glioma xenograft cells. A. Comet assay showing representative comet tail length observed in pMU and pMC transfected 4910 and 5310 glioma xenograft cells along with control and pSV samples. Magnification 40×, Bar = 20 µm. B. Representative bar graph showing comet tail length in pMU- and pMC-treated 4910 and 5310 glioma cells. Error bars indicate ±SD. * significant at p<0.05 Vs control. C. FACS analysis shows cell cycle distribution in pMU- and pMC-treated 4910 and 5310 glioma xenograft cells D. Bar graph shows representative percentage of apoptotic cells in pMU- and pMC-treated verses untreated glioma cells. Error bars indicate ±SD. * significant at p<0.05 Vs control. E. FACS analysis showing dot plot of gated γH2AX expression and DNA content in different phases of cell cycle in pMU- and pMC-treated 4910 glioma cells. F. After gating γH2AX expression, its expression in sub G_0_-G_1_, G_1_, S and G_2_-M phases was divided and shown in different shades of gray in pMU and pMC transfected cells compared to pSV. G. Bar graph showing number of cells expressing γH2AX in sub G_0_-G_1_, G_1_, S and G_2_-M phase in pMU- and pMC-treated 4910 glioma xenograft cells along with pSV. 10,000 cells were analyzed during each process. Error bars indicate ±SD. * significant at p<0.05 Vs control. H. Western blot analysis of γH2AX shows expression of γH2AX in pMU and pMC transfected 4910 and 5310 glioma cells along with control and pSV. GAPDH shows equal loading. Each experiment was repeated 3 times.

Further, PI staining demonstrated that pMU- and pMC-treated 4910 and 5310 cells exhibited significant increase in sub G_0_-G_1_ cells (apoptotic cells) (Figure 4C). 38–45% of cells were in the apoptotic phase in pMU- and pMC-transfected 4910 and 5310 human glioma xenograft cells as compared to <5% of control and pSV-treated cells (Figure 4D). To further evaluate the expression of γH2AX, Western blotting and FACS analysis were carried out. Increased expression of γH2AX was observed in both pMU- and pMC-treated 4910 and 5310 glioma cells compared to control and pSV (Figure 4H). Analysis of γH2AX expression and DNA content by FACS revealed an increased accumulation of γH2AX expression in G_1_, S, G_2_-M and sub G_0_-G_1_ in MU- and MC-treated glioma cells compared to pSV (Figure 4E). Figure 4F, shows the gated γH2AX expression divided into sub G_0_-G_1_, G_1_, S and G_2_-M phases of the cell cycle in different shades of grey colors after pMU- and pMC-treatment compared to pSV. The maximum accumulation of γH2AX expression was seen in the sub G_0_-G_1_ phase of pMU- and pMC-transfected 4910 glioma cells (p<0.05) (Figures 4G). Similarly, 5310 glioma treated cells expressed progressively increased levels of γH2AX in sub G_0_-G_1_ compared to pSV (data not shown).

Further, studies on inhibition of DNA PKcs by NU7441 (a DNA PKcs inhibitor) resulted in significant inhibition of proliferation as assessed by MTT and BrdU assay (Supplementary Figure S2A). FACS analysis indicated sub G_0_-G_1_ arrest in 4910 glioma xenograft cells treated with DNA PKcs inhibitor (Supplementary Figure S2B). Expression of γH2AX in 4910 cells with DNA PKcs, EGFR and CHK2 inhibitors alone and in combination with CHK2 inhibitor, showed increased levels of γH2AX compared to untreated cells (Supplementary Figure S2C). Supplementary Figure S2C depicts the prominent increase in the expression of γH2AX with the combined inhibition of DNA PKcs+EGFR+CHK2 compared to individual treatments. These result clearly demonstrates how pMU and pMC treatments orchestrate complex signaling in regulating key proteins leading to accumulation of DSBs. Taken together, these results indicate that induction of apoptosis after pMU and pMC treatments is due to accumulated unrepaired DSBs in 4910 and 5310 glioma cells compared to untreated cells.

### Expression of HIF-1α, γH2AX and RAD51 under hypoxia and in combination with irradiation (IR) after pMU and pMC treatments in glioma cells

GBM forms solid tumors, thus the cells at the core of the tumors become anaerobic due to hypoxia. Irradiation and chemotherapy fail to induce DNA damage in GBM cells thus may not result in DSBs and apoptosis. We have shown the effect of pMU and pMC shRNA on GBM cells under high oxygen levels (Normoxia) results in DSBs and apoptosis. Based on above facts, we further examined the efficiency of the pMU and pMC treatment under hypoxia along with irradiation (IR). 4910 and 5310 glioma cells showed clear change in cell morphology after hypoxic conditions (Supplementary Figure S3A). Cell proliferation assay using BrdU incorporation showed that pMU and pMC transfection significantly decreased proliferation of hypoxia alone, IR alone and hypoxia+IR exposed glioma cells compared to the respective controls in 4910 glioma cells (Supplementary Figure S3B). We observed that glioma cells, when treated with pMU and pMC constructs under normoxia, hypoxia, normoxia+IR and hypoxia+IR reduced the expression and activity of hypoxia inducing factor 1 alpha (HIF-1α), when compared with pSV and respective controls in both 4910 and 5310 glioma cells (Figure 5D and Supplementary Figure S3C).

**Figure 5:** Effect of pMU and pMC treatments on γH2AX (NHEJ) and Rad51 (HR) expression in hypoxia alone , irradiation (IR) alone and hypoxia+IR exposed glioma cells. A. FACS analysis shows cell cycle distribution in pMU- and pMC-treated hypoxic, IR and hypoxic+IR exposed 5310 glioma xenograft cells. 5,000 cells were analyzed during each process. Number(%) represent respective apoptotic cell population in samples. B. FACS analysis showing dot plot of gated γH2AX expression after pMU and pMC transfection in hypoxic, IR and hypoxic+IR exposed 5310 glioma xenograft cells along with pSV and control. C. Bar graph showing number of cells expressing γH2AX in sub G_0_-G_1_, G_1_, S and G_2_-M phase in pMU- and pMC-treated hypoxic, IR and hypoxic+IR exposed 4910 and 5310 glioma xenograft cells along with pSV and control. D. Western blot analysis of γH2AX shows expression of HIF-1α, γH2AX and Rad51 in pMU and pMC transfected hypoxic, IR and hypoxic+IR exposed 5310 glioma cells along with pSV and control. GAPDH served as loading control. E. Immunocytochemistry analysis was carried out to show formation of γH2AX and Rad51 foci in pMU- and pMC-treated hypoxic, IR and hypoxic+IR exposed 4910 glioma xenograft cells along with control and pSV. Each experiment was repeated 3 times.

We determined extent of DNA fragmentation post-transfection by TUNEL assay. In TUNEL assay, increased TUNEL-positive cells were observed in pMU and pMC-transfected hypoxia, normoxia+IR and hypoxia+IR glioma cells compared to respective controls (Supplementary Figure S3D). The number of apoptotic cells were counted post-transfection and the percentage of TUNEL positive apoptotic cells was plotted (Supplementary Figure S3E). the apoptotic cells were significantly higher in pMU- and pMC-transfected hypoxia, normoxia+IR, hypoxia+IR cells when compared to pSV and respective controls (Supplementary Figure S3E). In addition, to confirm the accumulation of DSBs primary to apoptosis induction in pMU- and pMC-treated glioma cells, we detected the γH2AX and PI expression by FACS analysis in hypoxia, normoxia+IR and hypoxia+IR glioma cells after pMU and pMC transfection. We found elevated γH2AX expression in apoptotic cells in pMU- and pMC-treated hypoxia, normoxia+IR and hypoxia+IR glioma cells compared to respective controls (Figure 5A, 5B and 5C). Elevation in γH2AX expression was further confirmed by Western blot analysis in pMU- and pMC-transfected hypoxia, normoxia+IR and hypoxia+IR cells compared to respective controls (Figure 5D). We noticed IR could induce the expression of γH2AX in glioma cells with G2-M arrest but it failed to induce the γH2AX expression under hypoxia in glioma cells (Figure 5D). FACS analysis showed transfection of hypoxia, normoxia+IR and hypoxia+IR glioma cells with pMU and pMC could readily elevate γH2AX expression and induce apoptosis in hypoxia, normoxia+IR and hypoxia+IR 4910 and 5310 glioma cells (Figure 5A, 5B and 5C). Moreover, there was increased expression of γH2AX expression in apoptotic cells compared to respective control samples (Figure 5C). These results further show how our constructs stabilized radiation induced DNA damage in hypoxia and induced apoptotic cell death.

Increased expression of Rad51 in hypoxic, normoxia+IR and hypoxia+IR glioma cells was markedly lowered by pMU and pMC treatments in glioma cells (Figure 5D). The above results were assessed by immunocytochemistry, wherein increased γH2AX foci were observed in pMU- and pMC-transfected glioma cells. In corroboration with Western blot analysis, lowered Rad51 foci was seen in pMU- and pMC-treated hypoxia, normoxia+IR, hypoxia+IR exposed glioma cells (Figure 5E). These results highlight that our constructs used in the study impair DNA repair efficiency not only under normoxia but also under hypoxia alone and in combination with IR. This finding is particularly interesting from a clinical standpoint for hypoxia favored radio- and chemo-resistant solid tumors.

### *In vivo* studies

Aggressive tumor formation was noticed in glioma xenograft injected mouse brains compared to normal brains. Further, Hematoxylin and Eosin staining performed on mouse brains revealed a prominent reduction of tumor growth in pMU- and pMC-treated mouse brains when compared to the controls [22], [26]. We next pursued to analyze the expression of DDR related proteins in control, pMU and pMC-treated brain sections. Immunohistochemical analysis of these brain sections from all the groups showed decreased expression of DNA PKcs and ATM after pMU and pMC treatments compared to controls (Figures 6A and 6B). We also noticed a prominent increase in the expression of γH2AX in pMU- and pMC-transfected cells compared to controls (Figure 6C). These *in vivo* results substantiated our *in vitro* results.

**Figure 6:** Immunohistochemistry analysis of paraffin embedded tissue sections prepared from nude mice implanted orthotopically with glioma cells and treated with pMU and pMC. IHC analysis shows expression of DNA PKcs (A), ATM (B) and γH2AX (C) in both pre-established 4910 and 5310 glioma tumors treated with pMU and pMC constructs. Magnification 60×. Bar = 20 µm. Each experiment was repeated 3 times.

## Discussion

GBM has various genetic deletions, amplifications and point mutations that lead to the activation of signal transduction pathways involving cell survival and DNA repair pathways [30]. DNA PK is a nuclear serine/threonine protein kinase involved in NHEJ, DNA repair and V (D) J recombination. Ku70, Ku80 and DNA PKcs form the DNA PK complex. Ku's high specificity to interact with DNA ends of DSBs initiates the recruitment of DNA PKcs. Over-expression of DNA repair proteins in GBM elevate efficiency of these cancer cells to repair DNA damage making treatment of GBM inherently difficult. Reduced DNA repair mechanism and/or induction of apoptosis are the possible interventions to inhibit proliferation of cancer cells including glioma. Therefore, in the present study, we focused on the DNA damage response of glioma cells after pMU and pMC treatments. We demonstrated that transcriptional silencing of MMP9 in combination with uPAR/cathepsin B inhibited proliferation of glioma cells compared to controls.

We observed a prominent decrease in the expression of NHEJ repair machinery proteins after pMU and pMC treatments. Ku70 and Ku80 DNA binding activity after pMU and pMC treatments were decreased compared to controls. These results clearly suggest that the initial Ku binding to DSBs, which is a critical step for recruitment of DNA PKcs in NHEJ repair response is inhibited by pMU or pMC treatments. Reduced phosphorylation of DNA PKcs T^2609^ in pMU- or pMC- treated glioma cells further strengthens these results and the earlier reported findings, wherein, decreased DNA end processing of DSBs was observed by inhibition of DNA PKcs T^2609^ phosphorylation [31].

To gain further insight into the mechanism by which these constructs retard DNA repair efficiency, we investigated the signal cascade involved in the regulation of DNA PK activity. Ku80 participates in cellular response to external stimuli and also the subcellular localization of Ku is controlled by a variety of external growth regulating stimuli [32], [33]. Integrins play a key role in cell adhesion to ECM. Interaction of integrins with ECM transduces signals for cell proliferation, adhesion, migration and angiogenesis. Earlier studies showed co-immunoprecipitation of the β1 integrin with uPAR [34]. Our present study results show complex formation of β1 integrin with uPAR, MMP-9 and cath B on cell surface, as confirmed by immunoprecipitation. Cav-1 has been shown to co-immunoprecipitate with the β1 integrin and uPAR [35]. Signaling mediated by this complex can also involve EGFR [36]. These results demonstrate the complex interplay among MMP9, uPAR, cathepsin B, β1 integrin and EGFR in regulating DNA PK activity. cSrc/cav-1 mediated nuclear EGFR internalization is associated with activation of DNA PK [37]. As expected, expressions of integrins, caveolin 1, cSrc, which are involved in the perinuclear transport of EGFR were reduced. Further, immunoprecipitation analysis demonstrated decreased EGFR association with DNA PKcs, Ku70 and Ku80 after pMU or pMC treatments in glioma cells. Moreover, nuclear expression of EGFR was associated with elevated DNA repair response. In agreement with the earlier reported data, we also noticed a reduction in the nuclear expression of DNA PKcs, Ku70, Ku80 and EGFR. These findings strengthen the involvement of extracellular signaling mediated through β1 integrin-EGFR signaling resulted in reduced DNA PK activity, which is important for the NHEJ-mediated repair mechanism in glioma cells.

In order to assess the relationship between DNA damage signaling by pMU or pMC treatments and HR repair pathway, ATM, a protein kinase critical for the response to DNA DSBs, was assessed [38], [39]. RAD51 related proteins acting downstream of ATM is required to ensure high fidelity of DNA repair by using an undamaged homologous DNA template to synthesize the damaged DNA strand [40]. Unrepaired DNA damage could activate cell-cycle checkpoints to allow sufficient time to repair damage or alternately, depending on the extent of damage, a signal may be transduced that initiates a signal cascade leading to a permanent growth arrest or apoptosis [41]–[43]. Genetic alteration of the CHK2 phosphorylation site rendered cells deficient in DSB repair [44]. As expected, we have noticed a prominent reduction of ATM, RAD51 and pCHK2 in glioma cells after pMU and pMC treatments. In addition, expression of survival signaling proteins pERK, AKT and pAKT were also prominently reduced.

It has been shown that DSBs, if left unrepaired, will lead to cell death [41]. Not only was the role of Ku established in the NHEJ repair mechanism, but it was also shown that depletion of Ku80 was associated with increased incidence of DNA DSBs, chromosome aberrations and shortening of telomere ends. Downregulation of Ku80 has been shown to suppress spontaneous tumors by induction of apoptosis [45]. Based on all these observations, we thought that the anti-proliferative effect of pMU and pMC treatments could be due to accumulated unrepaired DSBs, resulting in apoptosis. Hence, we investigated the existence of DSBs by observing the presence of γH2AX foci in pMU- and pMC-treated glioma cells. γH2AX has been associated with induction of apoptosis [46] and it is also proposed that γH2AX foci correlate with the number of DSBs with a 1∶1 ratio. In agreement with these earlier findings, we noticed an increase in comet tail length and γH2AX expression in different phases of the cell cycle, with a maximum percentage of γH2AX positivity in the sub G_0_-G_1_ phase, which indicates the induction of apoptosis in cells with accumulated DSBs after pMU and pMC treatments. Our inhibitory studies showed a marked increase in γH2AX expression when DNA PKcs/EGFR/pCHK2 were inhibited together, which shows the selective advantage of our constructs in inducing apoptosis by DSB accumulation and by regulating the DNA damage response machinery by different signal transduction pathways.

Solid tumors including GBM has lowered median pO_2_ levels (hypoxia) at the core of the tumor compared to surrounding normal tissue and hypoxia favors glioma tumor progression [47]–[49]. DNA radicals generated from radiation must react with oxygen to form organic peroxides that stabilize the radiation induced DNA damage [4]. Another important factor for radiation resistance by glioma cells is its enhanced DNA repair mechanism. In the case of chemotherapy resistance, the state of hypoxia itself and distance of the tumor cells from the blood vessel makes the tumor cells less effective to chemotherapeutic drugs [50]–[52]. Strategies carried out to exploit tumor hypoxia had some positive outcome in other cancers, however it was ineffective in GBM [53], [54]. Any intervention at the cellular level could lead to potentially better therapeutic options for GBM treatment. Our results demonstrate that silencing of MMP9 in combination with uPAR/cathepsin B, which are over expressed in gliomas, affects the expression of γH2AX (NHEJ), RAD51 (HR) and lowers the activity of HIF-1α. This signaling downregulates the repair mechanism and sensitizes the glioma cells to undergo apoptosis under normoxia, hypoxia and in combination with IR. We observed hypoxia, normoxia+IR and hypoxia+IR glioma cells over-expressed RAD51 compared to control. This shows how hypoxia and IR could elevate the expression of repair genes. One of the interesting findings of our study is the stabilization of IR-induced DNA damage under hypoxia by pMU and pMC treatments. This finding is potentially important because normally IR therapy fails to induce DNA damage under hypoxia; these findings are further supported by reduced DNA damage response. In addition to *in vitro* results, we also observed reduced expression of DNA PKcs and ATM proteins *in vivo* in xenograft cells after pMU and pMC treatments compared to control brain tumor sections.

Resistance to apoptosis and increased survival signaling are the major contributors for cancer cell survival. Drugs that target both of these pathways would provide a greater therapeutic benefit for cancer patients. Our earlier *in vitro* and *in vivo* studies showed a promising outcome with bicistronic constructs in the treatment of glioma by induction of apoptosis in cancer cells. The present study revealed for the first time that silencing MMP9 in combination with either uPAR or cathepsin B orchestrates a complex signal cascade to regulate both NHEJ and HR pathways, which are involved in DSB repair. The suppression of the DNA damage repair mechanism by these constructs leads to an increase in the levels of un-repaired DNA lesions where the cell overcomes the survival signaling by EGFR/AKT and ERK pathways to undergo apoptosis. Our study clearly demonstrated the potential anti-proliferative effect of bicistronic constructs pMU and pMC by reducing repair of DNA damage and inducing apoptosis. Given the genetic heterogeneity of cancer cells, targeting the gene products, which have multi-target potential, with similar beneficial effects under a different tumor microenvironment may prove to be a better therapeutic method to treat glioma.

## Materials and Methods

### Ethics statement

The Institutional Animal Care and Use Committee of the University of Illinois College of Medicine at Peoria, Peoria, IL, USA, approved all surgical interventions and post-operative animal care. The consent was written and approved. The animal protocol number is 851, dated April 23, 2009, and renewed on March 15, 2011.

### Cell lines and chemical reagents

Glioblastoma xenograft cells (4910 and 5310), kindly provided by Dr. David James of the University of California, San Francisco, were generated and maintained in mice and were highly invasive in the mouse brain. At 3–4 passages of xenograft cells from mice, heterotrophic tumors were frozen and these frozen stocks were used for further experimental studies up to the 10^th^ passage to obtain consistent results. Xenograft cells were maintained in RPMI 1640 supplemented with 10% FBS (Invitrogen Corporation, Carlsbad, CA), 50 units/mL penicillin and 50 µg/mL streptomycin (Life Technologies, Inc., Frederick, MD). Cells were maintained in a 37°C incubator with a 5% CO_2_ humidified atmosphere. For hypoxia induction, cells were incubated at 1.0% oxygen for 24 hours. 24 hours post-transfection, cells were irradiated at a single (8 Gy) dose of radiation using the RS 2000 Biological Irradiator (Rad Source Technologies, Inc., Boca Raton, FL), which was operated at 150 kV/50 mA for the radiation treatments, and cultured for additional 24 hours. We used the following antibodies in the present study: DNA PKcs, pDNA PKcs (T^2609^), Ku70, Ku80, EGFR, Caveolin-1, ATM, ATR, CHK2, pCHK2, γH2AX, SP1, AKT, pAKT, ERK, pERK, β1 integrin, MMP9, uPAR, cathepsin B and glyceraldehyde-3-phosphate dehydrogenase (GAPDH) (all from Santa Cruz Biotechnology, Santa Cruz, CA), pATM, pATR and pBRCA (Cell Signaling, Danvers, MA). Species-specific secondary antibodies conjugated to HRP, Alexa Fluor 488, and Alexa Fluor 595 (Invitrogen, Carlsbad, CA) were used in this study. All transfections were carried out using FuGene HD transfection reagent according to the manufacturer's instructions (Roche Applied Science, Madison, WI).

### Construction of shRNA expressing plasmids, transfection conditions and inhibitor treatment

Plasmid constructs containing bicistronic shRNAs pMU, pMC and scrambled vector (pSV) with an imperfect sequence designed in our laboratory [22], [23] were used to transfect the xenograft cells. Cells were transfected with either plasmid-expressing shRNA against pMU, pMC or pSV at 70–80% confluence for 48 hours. For the inhibitor study, cells seeded in a six-well plate were treated for 24–48 hours with NU7441 (1–10 µM), a potent DNA PKcs inhibitor, GW2974 (0.5 µM), a potent inhibitor of EGFR, and NSC 109555 ditosylate (0.2 µM), a selective CHK2 inhibitor.

### Cell proliferation and cell cycle analysis

Cell growth rate was determined using MTT assay ([3-(4, 5-dimethylthiazol-2-yl)-2, 5-diphenyltetrazolium bromide]; Sigma Aldrich, St. Louis, MO) as described previously [55]. BrdU incorporation assay was performed (Roche Diagnostics, Indianapolis, IN), according to the manufacturer's instructions. Clonogenic assay was carried out by seeding 500 cells in 100 mm plates after the transfection described above, and survival fraction was calculated based on the colony forming ability of cells after 2 weeks. Fluorescence activated cell sorting (FACS) analysis was done after 48 hours of transfection as described previously [56]. FACS analysis was done on at least 10,000 cells from each sample and cell cycle data were analyzed using a FACS Calibur Flow Cytometer (BD BioSciences, San Jose, CA). FACS analysis for γH2AX expression and propidium iodide (PI) staining in different phases of cell cycle were carried out by incubating trypsinized cells with primary antibody (1∶10 ratio) for 1 hour at 37°C followed by secondary antibody treatment for 30 minutes.

### Reverse transcription polymerase chain reaction (RT-PCR)

Total RNA was extracted from transfected cells using TRIZOL reagent (Invitrogen, CA) according to standard protocol. RNA (1 µg) was used as a template for reverse transcription reaction (Roche Applied Science, Indianapolis, IN), followed by PCR analysis. We used the following sequences for the forward and reverse primers: DNA PKcs: 5′GCCTTAGCACATGCAGATGA 3′ (forward) and 5′ GCCACTTGACCAGATCCAAT 3′ (reverse); Ku70: 5′ATGGCAACTCCAGAGCAGGTG 3′ (forward) and 5′AGTGCTTGGTGAGGGCTTCCA 3′ (reverse); Ku80: 5′ TGACTTCCTGGATGCACTAATCGT3′ (forward) and 5′TTGGAGCCAATGGTCAGTCG 3′ (reverse) and GAPDH: 5′AGCCACATCGCTCAGACACC 3′ (forward) and 5′GTACTCAGCGGCCAGCATCG 3′ (reverse).

Reverse transcriptase PCR was set up using the PCR cycle [95°C for 5 min, (95°C for 30 sec, 55–60°C for 30 sec, and 72°C for 30 sec)×30 cycles, 72°C for 10 min]. PCR products were resolved on a 1.6% agarose gel, visualized, and photographed under UV light.

### Immunoblotting and immunoprecipitation assay

For Western blot analysis, equal amounts of protein fraction were resolved over SDS-PAGE along with standard protein marker and immunoblotted with primary antibody followed by HRP-conjugated secondary antibodies. Signals were detected using the ECL Western blotting detection system (Pierce, Rockford, IL). *IgG served as negative control for all the immunoblot analysis*. The specificity of the proteins evaluated by Western blotting were verified based on its molecular weight as mentioned in manufacturer's data sheet and evaluated it against the standard protein marker (Precision Plus Protein™ Kaleidoscope Standards, Bio-Rad, Hercules, CA). Immunoprecipitation assays were carried out by incubating a minimum of 100–500 µg total cell lysate with antibody overnight at 4°C on a rotating shaker. Protein A/G agarose beads (Miltenyi Biotec, Auburn, CA) were added to the above complex and incubated for 1 hour on ice. Immunoprecipitates were eluted using µMac columns according to the manufacturer's instructions and were immunoblotted with appropriate primary and secondary antibodies.

### Subcellular fractionation

Cytoplasmic and nuclear fractions were prepared using an Active Motif Nclear Extraction Kit according to the manufacturer's instructions (Active Motif, Carlsbad, CA). Harvested cells were lysed in hypotonic buffer for 30 min at 4°C and centrifuged. The supernatant was collected as the cytosolic fraction. The nuclear pellet was re-suspended in complete lysis buffer for 30 min at 4°C and the nuclear fraction was collected after centrifugation. Immunoblot analysis was performed for DNA-PKcs, Ku70, Ku80, EGFR, and lamin B (served as loading control) in the nuclear fractions. The purity of nuclear extracts was confirmed by absence of cytoplasmic marker α-tubulin as assessed by Western blotting (data not shown).

### KU70/80 DNA binding activity

Binding efficiency of Ku70 and Ku80 to DSBs was quantified using a Ku70/Ku80 Active Motif DNA Repair Kit (Carlbad, CA) according to manufacturer's instructions. Nuclear protein (1.25–2.5 µg) was loaded onto oligonucleotide coated 96-well plate and incubated for 1 hour at room temperature. Ku70 or Ku80 antibodies were added to the wells and incubated for 1 hour. The binding of Ku to the DSBs was measured spectroscopically at 450 nm absorbance.

### Immunofluorescence

Cells grown in two-well chamber slides were washed with PBS, fixed with ice-cold methanol and permeabilized with 0.3% triton X followed by blocking with 2% BSA in PBS. Cells were incubated with primary antibodies or IgG (specific to the subclass of primary antibody) for either 2 hours at room temperature or overnight at 4°C, washed with PBS, and incubated with Alexa Fluor® conjugated secondary antibodies for 1 hr at room temperature. Nuclei were counterstained with DAPI and analyzed under a microscope (Olympus BX61 Fluoview, Minneapolis, MN). IgG served as negative control.

### Comet Assay

Cellular DNA damage was evaluated using a Comet Assay Kit (Cell Biolabs' OxiSelect™ STA-350) according to the manufacturer's instructions. Comet tail indicating degree of double strand DNA damage accumulation was measured against intact DNA. Results were quantified and normalized to control.

### Hypoxia inducible factor - 1 (HIF-1) DNA binding assay

The extracted nuclear fractions described above were used for the HIF-1 DNA binding assay. HIF-1 binding efficiency to the hypoxia responsive elements was analyzed using a Trans-AM HIF Transcription Factor Assay Kit (Active Motif, Carlsbad, CA). The assay kit contains a 96-well plate coated with oligonucleotide containing the HIF-1 binding site from the EPO gene. Active HIF-1 contained in cell extracts selectively binds to this oligonucleotide and can be revealed by incubation with antibodies using enzyme-linked immunosorbent assay technology with absorbance reading. Approximately 10 ug of nuclear extract was used and analyzed for HIF-1 binding activity following manufacturer's instructions.

### *In situ* terminal deoxynucleotidyl transferase dUTP nick end labeling (TUNEL) assay

The apoptotic cell death population of all treated cells from 4910 and 5310 glioma cells was detected using a TUNEL Apoptosis Detection Kit (Roche Diagnostics, Indianapolis, IN) following manufacturers protocol. Cells were incubated in the TUNEL reaction mixture at 37°C for 1 hour and further visualized for the incorporated fluorescein under confocal microscope. Positive control of the TUNEL assay was confirmed by incubating fixed and permeabilized cells with DNase I for 10 min at room temperature to induce DNA strand breaks, prior to labeling procedures. Negative control of the TUNEL assay was confirmed by incubating fixed and permeabilized cells in label solution (without terminal transferase) instead of TUNEL reaction mixture.

### Immunohistochemistry

Both 4910 and 5310 glioma xenograft cells were injected intracerebrally into nude mice with a 10 µl aliquot (0.2×10^5^ cells/µl) under isofluorane anesthesia with the aid of a stereotactic frame. Tumors were allowed to grow for 10 to 12 days, and the animals were separated into groups (six animals per group). Alzet mini pumps were implanted for pMMP-9 delivery at the rate of 0.2 µl/h. The concentration of the plasmid solution was 2 µg/µl (100 µl per mouse, six mice in each group). After five weeks or when the control animals started showing symptoms the mice were sacrificed by intracardiac perfusion, first with PBS and then with 4% paraformaldehyde in normal saline. The brains were collected, stored in 10% buffered paraformaldehyde, processed, embedded in paraffin, and sectioned (5 µm thick) using a microtome from control and treatment groups. Further, deparaffinization was done following standard protocol. Antigen retrieval was performed by treating the sections with citrate buffer at 95 degrees for 15–20 minutes followed by hydrogen peroxide treatment for 30 minutes. The sections were rinsed with PBS and blocked with 1% BSA in PBS to prevent non-specific staining and further incubated with primary antibodies (1∶50 dilution) at 4°C overnight. The sections were then incubated either with HRP-conjugated or Alexa Fluor conjugated secondary antibody for 1 h at room temperature and followed by 3,3 – diaminobenzidine (DAB) or 4,6-diamino-2-phenylindole (DAPI) solution incubation for 30 min. The sections were counterstained with hematoxylin to visualize the nucleus. Slides were mounted and photographed with a CCD camera attached to a microscope.

### Statistical analysis

All data are presented as mean ± standard deviation (SD) of at least three independent experiments. Statistical comparisons were performed using Graph Pad Prism software (version 3.02). Bonferroni's post hoc test (multiple comparison tests) was used to compare any statistical significance between groups. Differences in the values were considered significant at *p*<0.05.

## Supporting Information

Figure S1 **Anti-proliferative effect of pMU and pMC in 4910 and 5310 human glioma xenograft cells.** A. BrdU incorporation assay carried out in both glioma cells in pMU and pMC-treated cells compared to control and pSV (p<0.05) Vs control. B. Survival fraction was calculated based on colony forming ability of transfected 4910 and 5310 glioma cells in pMU and pMC treated cells compared to untreated. Each experiment was repeated 3 times. Error bars indicate ±SD. * significant at p<0.05 Vs control. C. Immunocytochemistry analysis shows expression of EGFR in pMU and pMC treated 4910 glioma xenograft cells. Green signal indicate EGFR expression and nucleus is stained with DAPI. Magnification 60×, Bar = 20 µm. Each experiment was repeated 3 times.
(TIF)

Figure S2 **Anti-proliferative role of DNA PKcs inhibition in 4910 and 5310 glioma xenograft cells.** A. MTT and BrdU assay. MTT assay shows dosage effect of DNA PKcs inhibitor-NU7441 in 4910 glioma xenograft cells. BrdU incorporation assay shows effect of inhibition of DNA PKcs in 4910 glioma xenograft cells. Error bars indicate ±SD. * significant at p<0.05 Vs control. B. FACS analysis showing effect of DNA PKcs inhibitor (NU7441) in 4910 glioma xenograft cells compared to DMSO control. Each experiment was repeated 3 times. C. Western blot showing expression of γH2AX after treatment with DNA PKcs, EGFR and CHK2 inhibitors alone and in combination in 4910 glioma cells compared with DMSO and control. GAPDH shows equal loading.
(TIF)

Figure S3 **Effect of pMU- and pMC-treated hypoxic, IR and hypoxia+IR exposed glioma xenograft cell.** A. 4910 and 5310 cell morphology observed in normoxic and hypoxic conditions. B. BrdU incorporation assay carried out in hypoxic, IR and hypoxia+IR exposed 4910 glioma cells represent significant reduction in proliferation of glioma cells in pMU and pMC-treated cells compared to pSV and control (p<0.05). C. HIF-1α DNA binding assay performed by using Active motif kit shows HIF-1α protein binding to oligonucleotide in pMU- and pMC- treated 4910 and 5310 hypoxic, IR and hypoxia+IR exposed glioma xenograft cells along with pSV and control. Error bars indicate ±SD. * significant at p<0.05 Vs control. D. TUNEL assay showing TUNEL positivity in pMU and pMC treated hypoxic, IR and hypoxia+IR exposed 4910 glioma cells compare to pSV and control. E. Bar graph showing percentage of TUNEL positive cells in pMU- and pMC-treated hypoxic, IR and hypoxic+IR exposed 4910 and 5310 glioma xenograft cells along with pSV and control. Error bars indicate ±SD. * significant at p<0.05 Vs control.
(TIF)
